# Numerical study of the thermally stratified hemodynamic nanofluid flow with variable viscosity over a heated wedge

**DOI:** 10.3389/fchem.2022.1021303

**Published:** 2022-10-11

**Authors:** Noreen Sher Akbar

**Affiliations:** DBS&H, CEME, National University of Sciences and Technology, Islamabad, Pakistan

**Keywords:** magnetohydrodynamics, nanofluids, Runge–Kutta method, static and moving wedge, skin friction coefficient

## Abstract

We analyze the steady laminar incompressible boundary-layer magnetohydrodynamic impacts on the nanofluidic flux over a static and mobile wedge in the existence of an applied magnetic field. The Falkner–Skan wedge flow model is taken into consideration. Reynolds’ model is considered to introduce temperature-dependent viscosity. As in real life, most fluids have variable viscosity. The executive partial differential equations are converted into a set-up of ordinary differential equations by means of a similarity conversion. Numerical solutions are computed for the converted set-up of equations subjected to physical boundary conditions. The specific flow dynamics like velocity profile, streamlines, temperature behavior, and coefficient of local skin friction are graphically analyzed through numerical solutions. It is concluded that the laminar boundary-layer separation from the static and moving wedge surface is altered by the applied external electric field, and the wedge (static or moving) angle improves the surface heat flux in addition to the coefficient of skin friction. Furthermore, it is found that the methanol-based nanofluid is a less-efficient cooling agent than the water-based nanofluid; therefore, the magnitude of the Nusselt number is smaller for the water-based nanofluid. It is also observed that the addition of only 1% of these nanoparticles in a base fluid results in an enhancement of almost 200% in the thermal conductivity.

## Introduction

The fluid mechanical aspects of the boundary layer on the static and mobile wedges (Falkner–Skan flow) have received a lot of attention from researchers and scientists of fluid mechanics mainly because of their applications in diverse situations such as natural flow, mechanical flow, biological flow, and transport of fluids in industries. The laminar boundary-layer flow impacts for a fixed wedge engaged in the viscous incompressible fluid were first reported by Falkner and Skan (1931). It was the extension of Prandtl’s concept on the applications of boundary layers. In the review of the laminar boundary-layer flow over a wedge set at an angle ( m π ), where the flow in the direction of the wedge is represented by m >0 and the flow opposite to the wedge direction is represented by m <0 and m=0 , the Falkner and Skan problem reduces to the Blasius problem (i.e., flow through a wedge shape reduces to flow through a flat plate). They have used similarity transformation to convert the set-up from partial to ordinary differential equations. Thereafter, this work has been extended by many researchers (Tuncer and Keller, 1971; Tsung and Lin, 1987; Asaithambi, 1997; Hsing et al., 1997; Yih, 1998; Zaturska and Banks, 2001; Kuo, 2005; Ishak et al., 2006; Hartree, 2008). Hartree (2008) conveyed the numerical computations on the flow dynamics over a wedge. Tuncer and Keller (1971) numerically interpreted the boundary-layer problem of Falkner–Skan by means of a parallel shooting technique. Tsung and Lin (1987) investigated the laminar forced convection heat transfer over a wedge and discussed the effects of the Prandtl number. Asaithambi (1997) provided solutions to the Falkner–Skan problem by means of the finite difference numerical technique. Hsing et al. (1997) interrogated the characteristics of heat convection and fluid flow for the second-grade fluids over the wedge. Yih (1998) reported the forced convection effects on the boundary-layer flow over a wedge and discussed the uniform suction and blowing effects. Zaturska and Banks (2001) provided novel solution works for different ranges of wedge angle parameters (i.e., 37.844 < *β* < ∞, *β* = 37.844, 14.533<*β* < 37.844, 1<*β* < 14.533, and *β* = 1). Kuo (2005) applied a differential transform method (DTM) to solve the boundary-layer flow problem over a wedge and discussed the velocity and shear-stress fields. In continuation of the aforementioned studies on flow dynamics for a fixed and mobile wedge, Ishak et al. (2006) extended for micropolar fluids; Yang and Lan (2007) for velocity and shear-stress functions; Matsson (2008) for suction and blowing; Yang and Lan (2011) for the non-existence of the reversed flow; and Tiegang et al. (Fang et al., 2012) with algebraic decay consideration on the Falkner–Skan flow.

The motivation behind the huge intriguing research on the topic of nanofluids in recent years is due to an open range of practical applications in both the engineering and pharmaceutical industries. The dispersion of nano-scale particles in a base fluid provides the combination of the nanofluid and in most cases nanotubes, nanofibers, nanosheets, nanowires, or droplets being used for this purpose. It is experimentally (Murshed et al., 2005; Wang and Mujumdar, 2007; Yu and Xie, 2012; Mahian et al., 2013; Bianco et al., 2015) proved that the addition of only 1% of these nanoparticles in a base fluid results in an enhancement of almost 200% in the thermal conductivity. Some of the most recent applications of nanofluids are reported by Tripathi and Bég (2014) and Akbar et al. (2016a). The carbon nanotube (CNT) is one of the nanoparticles which can be dispersed in base fluids, and it has a wide range of applications in various disciplines. The dispersion of the CNT in base fluids and its effects on the enhancement of thermal conductivity were analyzed through an experimental study performed by Kim and Peterson (2007). They observed that the addition of only 1% SWNT results in a thermal conductivity increase of 10%, while only 3.5% was achieved in the case of aluminum oxide. Some other experimental studies (Sastry et al., 2008; Garg et al., 2009) examining thermal conductivity and heat transfer performance are also reported. Furthermore, Kamali and Binesh (2010) presented a numerical study on fixed heat flux consequences of the addition of multi-wall nanotubes. They used the finite volume method (FVM) and considered the power law model of viscous fluids for base fluids. Most recently, Chai et al. (2016) used TEM imaging and FTIR analysis for the MWCNT structure and chemical compound. They have concluded that the hydrogenated oil containing multi-wall carbon nanotubes has a 9.8% increase in thermal conductivity at a concentration of 100 ppm, while an increase of 7.2% and 4.5% is noted at a concentration of 50 ppm and 25 ppm, respectively. There are many applications of MHD flows in the field of science and engineering. The combined effects of MHD and the nanofluid flow have huge applications in science, technology, and industries. Most recently, Chamkha (1996), Thameem Bash, Sivaraj, Takhar et al. (1999), Chamkha et al. (2006), Akbar et al. (2016b), Akbar et al. (2016), Akbar et al. (2016d), Animasaun et al. (2019), Kumaran et al. (2019), Thameem Basha et al. (2019), Ashraf et al. (2020), Basha et al. (2020), Hamad et al. (2022), and Rasool et al. (2022) reported the study of MHD, and the nanofluid flow is reported in the literature.

In all the aforementioned studies, the study of the nanofluid flow through a static and movable wedge is not reported. However, considering the immense count of practical applications in flow over the wedge, few investigators (Yacob et al., 2011a; Yacob et al., 2011b; Khan and Pop, 2013; Dennis et al., 2015; Khan et al., 2015) have reported. Yacob et al. (2011a) solved the Falkner–Skan problem by means of the Keller-box numerical technique for a fixed and mobile wedge, considering copper, titania, and alumina nanofluids. A higher coefficient of skin friction is observed for Cu–water than for other cases. In other studies, Yacob et al. (2011b) further extended their analysis by means of multiple numerical solution techniques like Keller box, shooting, and the Runge–Kutta–Fehlberg method. Khan and Pop (2013) investigated the boundary layer impacts on a mobile wedge with the nanofluid flow. Khan et al. (2015) extended their model by considering various effects like radiations, MHD, and chemical reactions on the boundary layer over a wedge. Daub et al. (Dennis et al., 2015) experimentally studied the effects of a mobile wedge on the shockwave boundary layer. Most recently, some important works (Javaherdeh and Ashorynejad, 2014; Malvandi et al., 2014; Sheikholeslami and Ganji, 2015; Kasmani et al., 2016; Madaki et al., 2016; Salama, 2016; Akram et al., 2020) have reported on the flow over the wedge moving in the second-grade nanofluid, highlighting the impacts of the Cu–water combination of nanofluids over a mobile wedge, the homotopy asymptotic technique for the Falkner–Skan flow problem. The fluid transport in composite membranes used in water desalination is presented in recent articles (Ezaier et al., 2022a; Ezaier et al., 2022b; Ezaier et al., 2022c)**.**

Motivated by the aforementioned studies and findings, we extend the work of Kuo (2005), Khan et al. (Yacob et al., 2011a), Yacob et al. (2011b)**,** and Khan and Pop (2013) for the static and movable wedge to study the heat transfer properties of different nanofluids, that is, the water-based copper nanofluid and methanol-based copper nanofluid. The viscosity of the fluid is assumed to be temperature-dependent, and the effect of the magnetic field is also included. Similarity transformation is used to change a set of PDEs to a set of ODEs; then, the Runge–Kutta method is employed for the numerical solution. A comparative analysis is presented between the results of the current study and the previously published literature in the limited cases in the tabular form, and it is shown that a good agreement with existing results is noted. This study is applicable in aerodynamics and hydrodynamics, especially in enhancing oil refinement, industrial usage in geothermal sciences, generators working on MHD principles, multiple bearings and pumps, control effects on boundary layers, etc.

## Formulation of the problem

The numerical computations are performed for the boundary-layer impacts on a fixed or a mobile wedge flow problem considering the nanofluids’ case of copper nanoparticles and two different base fluids, that is, methanol and water. The geometrical diagram of this wedge flow problem is presented in Figure 1. A thermal equilibrium condition is maintained for the nanoparticles, and a temperature-dependent viscosity is conceded. The free stream velocity is considered to be u(x) = U_∞_ x^m^, while the mobile wedge has a velocity u(x) = U_w_x^m^. The range of m value varies between 0 and 1. Here, the effect of the applied magnetic field of strength $B_{0}$ is considered, but the effect of the induced magnetic field and Hall currents are not taken into consideration due to the low-magnetic Reynolds number and the smaller frequency of atom–electron collision (Krishna and Chamkha, 2019; Krishna et al., 2020). The current problem is interpreted for a Cartesian system of coordinates.

**FIGURE 1:** Geometry of the physical problem.

The pertinent equations that govern this physical flow problem are given as (See Refs (Tsung and Lin, 1987; Ishak et al., 2006))

$$\frac{\partial u}{\partial x}+\frac{\partial v}{\partial y}=0,$$ (1)

$$u\frac{\partial u}{\partial x}+v\frac{\partial u}{\partial y}=U_{e}\frac{dU_{e}}{dx}+\frac{1}{\rho_{nf}}\frac{\partial }{\partial y}\left(\mu_{nf}\left(T\right)\frac{\partial u}{\partial y}\right)-\frac{\sigma B_{0}^{2}}{\rho_{nf}}\left(u-U_{e}\right),$$ (2)

$$u\frac{\partial T}{\partial x}+v\frac{\partial T}{\partial y}=\alpha_{nf}\frac{\partial^{2}T}{\partial y^{2}}+\frac{\mu_{nf}\left(T\right)}{{\left(\rho C_{p}\right)}_{nf}}{\left(\frac{\partial u}{\partial y}\right)}^{2}.$$ (3)

The relevant boundary conditions are imposed in the forms:

Static wedge

$$\begin{array}{c} u=0,\;v=0,\;T=T_{w},\;at\;y=0,\\ u=U_{e}\left(x\right),\;v\to 0,\;T\to T_{\infty },\;as\;y\to \infty . \end{array}\}$$ (4)

Moving wedge

$$\begin{array}{c} u=u_{w}\left(x\right)=ax,\;v=0,T=T_{w},\;at\;y=0,\\ u=U_{e}\left(x\right),\;v\to 0,\;T\to T_{\infty },\;as\;y\to \infty . \end{array}\}$$ (5)

The characteristics of the nanofluid model are taken (Kim and Peterson, 2007; Sastry et al., 2008; Garg et al., 2009; Kamali and Binesh, 2010; Akbar et al., 2016a; Chai et al., 2016) as follows:

$$\mu_{nf}=\frac{\mu_{0}e^{-\alpha \theta }}{{\left(1-\varphi \right)}^{2.5}},$$ (6a)

$$\alpha_{nf}=\frac{k_{nf}}{{\left(\rho c_{p}\right)}_{nf}},\rho_{nf}=\left(1-\varphi \right)\rho_{f}+\varphi \rho_{s},$$ (6b)

$${\left(\rho c_{p}\right)}_{nf}=\left(1-\varphi \right){\left(\rho c_{p}\right)}_{f}+\varphi {\left(\rho c_{p}\right)}_{s},\;$$ (6c)

$${\left(\rho \gamma \right)}_{nf}=\left(1-\varphi \right){\left(\rho \gamma \right)}_{f}+\varphi {\left(\rho \gamma \right)}_{S},$$ (6d)

$$k_{nf}=k_{f}\left(\frac{k_{s}+2k_{f}-2\varphi \left(k_{f}-k_{s}\right)}{k_{s}+2k_{f}+2\varphi \left(k_{f}-k_{s}\right)}\right).$$ (6e)

The following similarity variables are introduced to convert the problem into a set-up of ordinary differential equations as determined in Ishak et al. (2006):

$$\eta =\sqrt{\frac{\left(m+1\right)a}{2\nu_{f}}}y,\theta =\frac{T-T_{\infty }}{T_{w}-T_{\infty }},\psi =\sqrt{\frac{2\nu_{f}xU_{e}\left(x\right)}{m+1}}f\left(\eta \right),$$ (7)

Here, ψ denotes the stream function and can be interpreted as u = ∂ψ/∂y and v = −∂ψ/∂x.

The following viscosity model known as Reynold’s model is considered (Akbar et al., 2016b):

$$\mu_{f}\left(\theta \right)=e^{-\left(\alpha \theta \right)}=1-\left(\alpha \theta \right)+O\left(\alpha^{2}\right),$$ (8)

On substituting (6, 7, and 8) into (2) to (4) with boundary conditions (4 and 5), the converted set-up of ordinary differential equations is given as follows:

$$\frac{(1-\left(\alpha \theta \right)}{{\left(1-\varphi \right)}^{2.5}}f^{\prime \prime \prime }+\frac{-\alpha \theta^{\prime }f^{\prime \prime }}{{\left(1-\varphi \right)}^{2.5}}+\left[\left(1-\varphi +\varphi \frac{\rho_{s}}{\rho_{f}}\right)\left\{ff^{\prime \prime }+\left(\frac{2m}{m+1}\right)\left(1-f^{\prime 2}\right)\right\}+M^{2}\left(1-f^{\prime }\right)\right]=0,$$ (9)

$$\left(\frac{k_{nf}}{k_{f}}\right)\theta^{\prime \prime }+\mathrm{Pr}\left(1-\varphi +\varphi \frac{{\left(\rho c_{p}\right)}_{s}}{{\left(\rho c_{p}\right)}_{f}}\right)\left[\left(f\theta^{\prime }\right)+E_{c}\frac{(1-\left(\alpha \theta \right)}{{\left(1-\varphi \right)}^{2.5}}{\left(f^{\prime \prime }\right)}^{2}\right]=0.$$ (10)

Static Wedge

$$\begin{array}{c} f\left(0\right)=0,\;f^{\prime }\left(0\right)=0,\;f^{\prime }\left(\infty \right)=1,\\ \theta \left(0\right)=1,\;\theta \left(\infty \right)=0. \end{array}$$ (11)

Moving Wedge

$$\begin{array}{c} f\left(0\right)=0,\;f^{\prime }\left(0\right)=\lambda ,\;f^{\prime }\left(\infty \right)=1,\\ \theta \left(0\right)=1,\;\theta \left(\infty \right)=0, \end{array}$$ (12)

where $\mathrm{Pr}={\left(\mu c_{p}\right)}_{f}/k_{f}$ is the Prandtl number and $\lambda =U_{w}/U_{\infty }$ is the constant moving wedge parameter, β=2m/m+1 , which corresponds to β=Ω/π for a total wedge angle Ω .

The coefficient of skin friction $c_{fx}$ along the *x-*direction and $Nu_{x}$ Nusselt number is given as follows:

$$c_{fx}=\frac{\mu_{nf}\left(T\right)}{\rho_{f}u_{w}^{2}}{\left(\frac{\partial u}{\partial y}\right)}_{y=0},\;Nu_{x}=\frac{-xk_{nf}}{k_{f}\left(T_{w}-T_{\infty }\right)}{\left(\frac{\partial T}{\partial y}\right)}_{y=0}.$$ (13)

Eq. 13 in non-dimensional form is

$${\left({Re}_{x}\right)}^{1/2}c_{fx}=\frac{\mu_{f}\left(\theta \left(0\right)\right)f^{\prime \prime }\left(0\right)}{{\left(1-\varphi \right)}^{2.5}},{\left({Re}_{x}\right)}^{1/2}Nu_{x}=-\frac{k_{nf}}{k_{f}}\theta^{\prime }\left(0\right).$$ (14)

## Numerical illustration

The shooting technique is utilized to numerically compute the solutions of Equations 9, 10 with boundary conditions (11 and 12). This boundary value problem is initially transformed into an initial value problem; then, initial guesses are set up for $f^{\prime \prime }\left(0\right)$ and $\theta^{\prime }\left(0\right)$ . Finally, the Runge–Kutta technique of the fourth order is considered to numerically interpret the solutions. Mathematics software Maple is used for the simulation. A better approximation is achieved for the values of $f^{\prime \prime }\left(0\right)$ and $\theta^{\prime }\left(0\right)$ by utilizing the Secant method. A minimal step size of Δη=0.01 is considered with an accuracy of the fifth decimal place for a better convergence criteria.

## Graphical results and discussion

The numerical computations are performed to present the graphical illustrations (see Figures 2–10) of numerous intrigued parameters on the velocity outline, temperature formation, skin friction coefficient, $N_{u}$ , and streamlines. Table 1 shows the characteristics of the base fluid and nanoparticles. Table 2 and Table 3 are computed for skin friction for refined ﬂuid with α=0 and λ=M=0 dimensionless heat flux of the refined fluid with α=0 and λ=M=Ec=0 for multiple variables of the wedge ( m ). Table 2 depicts the present results compared to the outcomes of Yacob et al. (Hamad et al., 2022)**,** Khan and Pop (Rasool et al., 2022)**,** and Khan et al. (Animasaun et al., 2019), and in Table 2, the present outcomes are correlated with those of Kuo (Kuo, 2005), Khan et al. (Animasaun et al., 2019), and Khan and Pop (Rasool et al., 2022)**.** The outcomes of the present study are in good accordance with previous results.

**FIGURE 2:** **(A–C)** Velocity profiles corresponding to multiple nanofluidic fractions: **(A)** (*α*), **(B)** (*M*), and **(C)** (*m*).

**FIGURE 3:** **(A,B)** Temperature profiles corresponding to multiple nanofluidic fractions: **(A)** (*α*) and **(B)** (*M*).

**FIGURE 4:** **(A,B)** Temperature profiles corresponding to multiple nanofluidic fractions: **(A)** (*m*) and **(B)** (*Ec*).

**FIGURE 5:** **(A,B)**: Skin friction coefficient corresponding to different base fluids, that is, water and methanol for **(A)** (*M*). **(B)** (*α*).

**FIGURE 6:** **(A,B)** Skin friction coefficient corresponding to different base fluids, that is, water and methanol for **(A)** wedge parameter (*m*) and **(B)** moving wedge parameter ( λ).

**FIGURE 7:** **(A,B)** Nusselt number corresponding to different base fluids, that is, water and methanol for **(A)** viscosity parameter (*α*) and **(B)** Eckert number (*Ec*).

**FIGURE 8:** **(A,B)** Nusselt number corresponding to different base fluids, that is, water and methanol for **(A)** wedge parameter (*m*) and **(B)** Hartmann number (*M*).

**FIGURE 9:** **(A–C)** Streamlines with the variation of the moving wedge parameter (λ). Other parameters are *m* = 1, *M* = 2, and *α* = 0.3.

**FIGURE 10:** **(A–C)** Streamline graph of the variation of (*α*). Other parameters are *m* = 1 and *M* = 2.

**TABLE 1:** Experimental values for the base fluid and nanoparticles (Sajjan et al., 2022).

Physical property	Base ﬂuids		Nanoparticle
	Water	Methanol	Cu
ρ (kg/m^3^)	997	792	8,933
$c_{p}$ (J/kg-K)	4,179	2,545	385
k (W/m-K)	0.613	0.2035	401
$P_{r}$	6.2	7.38	—

**TABLE 2:** Comparative study on skin friction for α=0 and λ=M=0 .

*m*	$f^{\prime \prime }\left(0\right)$			
	Current analysis	Khan et al. (2015)	Khan and Pop (2013)	Yacob et al. (2011a)
0	0.46960	0.4696	0.4696	0.4696
1/11	0.65499	0.6550	0.6550	0.6550
1/5	0.80213	0.8021	0.8021	0.8021
1/3	0.92768	0.9277	0.9277	0.9277
1/2	1.03890	1.0389	1.0389	1.0389
1	1.23259	1.2326	1.2326	1.2326

**TABLE 3:** Comparative study on heat transfer for pure ﬂuids with α=0 and λ=M=Ec=0 .

*m*	$-\theta^{\prime }\left(0\right)$			
	Current analysis	Khan et al. (2015)	Khan and Pop (2013)	Kuo (2005)
0	0.87691	0.8769	0.8769	0.87673
1	1.12796	1.1280	1.1279	1.1147

The effects of nanoparticle volume fraction ( φ=0,0.1,0.2 ) on the velocity profile with the impact of the viscosity parameter ( α=0, 0.8 ), Hartmann number ( M=0,1.3 ), and wedge parameter ( m=0,0.5 ) are shown in Figures 2A–C. It is detected that the velocity figure diminishes with growing values of nanoparticle volume fraction. Figure 2A reveals that the velocity profile diminishes with an increase in the magnitude of the viscosity parameter. Figure 2B predicts that the velocity profiles diminish the growing effects of the magnetic field. This outcome is homogeneous to that of Sheikholeslami et al. (Kumaran et al., 2019) in which the impacts of the applied magnetic field on the velocity profile have been noted as “magnetic field has the tendency to slow down the movement of the fluid which decreases the velocity profile.” This similarity validates our present model. Figure 2C shows that the velocity profile contracts with the growing magnitude of the wedge parameter. Finally, it is concluded that the thickness of the boundary layer decreases with the increasing magnitude of ϕ , α , M, and λ .

The behaviors of the viscosity parameter ( α=0, 0.8 ), Hartmann number ( M=0, 3 ), wedge parameter ( m=0,1 ), and Eckert number ( Ec=0,1 ) on temperature profiles corresponding to various quantities of the nanoparticle volume ratio ( α=0,0.1,0.2 ) are presented in Figures 3A,B and Figures 4A,B correlatively. It is detected that maximum temperature occurs at zero transverse displacements and vice-versa. The temperature outline enhances with the growing magnitude of the nanoparticle volume fraction. Figure 3A illustrates that the temperature profile diminishes with an increase in the magnitude of the viscosity parameter. Figure 3B displays that the temperature profile diminishes with increasing M . Figure 4A presents that heat flux reduces with the upsurging magnitude of λ . The effect of Eckert number on the temperature profile is illustrated in Figure 4B, and it is observed that heat flux enhances with the upsurging magnitude of Eckert number. Furthermore, the thickness of the convection boundary layer increases with the increasing Eckert number.

The variations of distinct quantities on $C_{f}$ for the considered types of base fluids (methanol and water) are discussed through Figures 5A,B and Figures 6A,B **.** It is seen that $C_{f}$ is more in the case of methanol base fluids than in water base fluids. It can be discerned from Figure 5A that the magnitude of $C_{f}$ , the coefficient, is more for upsurging the effects of magnetic field, that is, ( M=0, 1, 2 ). Figure 5B shows the variation of the viscosity parameter ( α=0, 0.3,0.6 ) on $C_{f}$ , and it is detected that $C_{f}$ diminishes with increasing F061. The behavior of the wedge parameter ( m=0, 0.3,0.6 ) on $C_{f}$ is presented in Figure 6A, and it is noted that $C_{f}$ upsurges for the larger value of the wedge parameter. The influence of the moving wedge parameter ( λ=0, 0.3,0.6 ) on the skin friction coefficient is illustrated in Figure 6B. It is pointed out that $C_{f}$ reduces with the increasing magnitude of the moving wedge parameter from 0 to 0.6.

The characteristics of $N_{u}$ for the Falkner–Skan wedge flow of CNT nanofluids corresponding to the considered forms of base fluids methanol and water are shown in Figures 7A,B and Figures 8A,B accordingly. It is found that the Nusselt number is more for methanol nanofluids than for water nanofluids. Figure 7A depicts the consequences of the viscosity parameter ( α=0, 0.3,0.6 ) on $N_{u}$ , and there is an upsurge in the Nusselt number with the increasing magnitude of the viscosity parameter. Figure 7B is sketched for the Eckert number ( Ec=0,0.2,0.4 ) effects on the Nusselt number, and it is observed that $N_{u}$ is inversely proportional to the Eckert number. Figure 8A illuminates the variation in Nusselt number for the wedge parameter ( m=0, 0.1,0.2 ). Here, the Nusselt number is more for a greater value of the wedge parameter. The impacts of applied MHD on $N_{u}$ are depicted in Figure 8B, and it is predicted that $N_{u}$ reduces with the upsurging magnitude of M .

Streamlines are the key characteristics of the fluid flow which are mathematically found when the stream function is constant. For different values of stream function, the variation of stream lines is illustrated in Figures 9A–C and Figures 10A–C accordingly. The variation of the moving wedge parameter ( λ=−0.5, 0,0.5 ) at fixed values of other parameters (*m* = 1, *M* = 2, *α* = 0.3) on streamlines is presented through Figures 9A–C, and it is revealed that for –ve value of the moving wedge parameter, the streamline patterns are parabolic in range 0<x<0.5 and patterns are non-linear with horizontal and vertical asymptotes (both axes) in range x>0.5 . There is no parabolic pattern for the +ve value of the moving wedge parameter. The effects of the viscosity parameter ( α=0,0.4,0.8 ) at fixed values of other parameters (*m* = 1, *M* = 2) on streamline patterns are elucidated through Figures 10A–C. It is revealed that there is a parabolic pattern in the range 0<x<0.75 for the value of α=0 and in the range 0<x<0.5 for the value of α=0.4 and in the range 0<x<0.25 for the value of α=0.8 . It is finally interpreted that the parabolic nature of streamline patterns reduces with the increasing value of the viscosity parameter.

## Conclusion

The impacts of relevant variable parameters on the characteristics of the Falkner–Skan wedge flow of a temperature-dependent viscous effect with CNT nanofluids have been discussed. The concluding results are summarized as follows:

• The extent of the boundary layer reduces with an upsurging magnitude of ϕ , α , M, and λ .
• The extent of the thermal boundary layer expands by enhancing the value of ϕ , and Eckert number, however, decreases with the increasing value of the wedge parameter, and M .
• $C_{f}$ is more in the case of methanol base fluids than for water base fluids.
• $C_{f}$ is more for the large value of the Hartmann number and wedge parameter; however, opposite trends are pointed for the viscous parameter and moving wedge parameter.
• Nusselt number is more for methanol nanofluids than for water nanofluids.
• The Nusselt number is proportional to the viscosity parameter and wedge parameter; however, it is related in an inverse proportion to the Eckert number and Hartman number.
• The parabolic nature of streamlines reduces for the –ve value to +ve value of the moving wedge parameter, and it also decreases with the increasing value of the viscosity parameter.

## Data Availability

The original contributions presented in the study are included in the article/Supplementary Material; further inquiries can be directed to the corresponding author.

## Nomenclature

$u_{w}$: wall velocity $\left(ms^{-1}\right)$
$B_{0}$: the magnitude of magnetic field strength
α: Reynolds viscosity parameter (−)
**U**_**∞**_, U_w_: free stream and wedge velocity $\left(ms^{-1}\right)$
η: similarity parameter (−)
K: fluid thermal conductivity $\left(Wm^{-1}K^{-1}\right)$
ϕ: volume portion of nanoparticles (−)
M **Hartmann Number** (−) θ: Hartmann Number (−) θ temperature dimensionless representation (−)
x, y: coordinates (m)
$c_{f}$: base fluid heat capacitance $\left(J{Kg}^{-1}K^{-1}\right)$
$Nu_{x}$: Nusselt number (−)
$c_{p}$: nanoparticles’ heat capacitance $\left(J{Kg}^{-1}K^{-1}\right)$
P: pressure $\left(Nm^{-2}\right)$
μ: viscosity $\left(Kgm^{-1}s^{-1}\right)$
Pr: Prandtl number (−)
$\rho_{nf}$: nanofluid density $\left(Kgm^{-3}\right)$
q: heat flux $\left(Wm^{-2}\right)$
$\alpha_{nf}$: thermal diffusivity of the nanofluid $\left(m^{2}s^{-1}\right)$
$Sh_{x}^{n}$: local nanoparticle Sherwood number
ν: kinematic viscosity of the nanofluid $\left(m^{2}s^{-1}\right)$
u,v: velocity components $\left(ms^{-1}\right)$
$\mu_{nf}$: (T) nanoparticle temperature-dependent viscosity
T: local fluid temperature (K)
***k*_*f*_**: thermal conductivity of the base fluid $\left(Wm^{-1}K^{-1}\right)$
***T*_*w*_**: wall temperature (K)
***k*_*nf*_**: nanofluid thermal conductivity $\left(Wm^{-1}K^{-1}\right)$
β: Hartree pressure gradient parameter (−)
λ: fixed mobile wedge parameter (−)
